The article "Implementation of a Heart Disease Risk Prediction Model Using Machine Learning" was retracted in 2023. Reasons: unreliable results or conclusions; concerns about the data; concerns about the peer review; concerns about the citations.

# Implementation of a Heart Disease Risk Prediction Model Using Machine Learning

**DOI:** 10.1155/2022/6517716

**Published:** 2022-05-02

**Authors:** K. Karthick, S. K. Aruna, Ravi Samikannu, Ramya Kuppusamy, Yuvaraja Teekaraman, Amruth Ramesh Thelkar

**Affiliations:** ^1^Department of Electrical and Electronics Engineering, GMR Institute of Technology, Rajam, Andhra Pradesh, India; ^2^Department of Computer Science and Engineering, School of Engineering and Technology, CHRIST (Deemed to be University), Bangalore, Karnataka, India; ^3^Department of Electrical Computer and Telecommunications Engineering, Botswana International University of Science and Technology, Palapye, Botswana; ^4^Department of Electrical and Electronics Engineering, Sri Sairam College of Engineering, Bangalore City, India; ^5^Department of Electronic and Electrical Engineering, The University of Sheffield, Sheffield S1 3JD, UK; ^6^Faculty of Electrical & Computer Engineering, Jimma Institute of Technology, Jimma University, Ethiopia

## Abstract

Cardiovascular disease prediction aids practitioners in making more accurate health decisions for their patients. Early detection can aid people in making lifestyle changes and, if necessary, ensuring effective medical care. Machine learning (ML) is a plausible option for reducing and understanding heart symptoms of disease. The chi-square statistical test is performed to select specific attributes from the Cleveland heart disease (HD) dataset. Support vector machine (SVM), Gaussian Naive Bayes, logistic regression, LightGBM, XGBoost, and random forest algorithm have been employed for developing heart disease risk prediction model and obtained the accuracy as 80.32%, 78.68%, 80.32%, 77.04%, 73.77%, and 88.5%, respectively. The data visualization has been generated to illustrate the relationship between the features. According to the findings of the experiments, the random forest algorithm achieves 88.5% accuracy during validation for 303 data instances with 13 selected features of the Cleveland HD dataset.

## 1. Introduction

According to WHO data, heart disease is the leading cause of mortality globally, resulting in 17.9 million deaths annually [1]. The most behavioural risk factors for cardiovascular disease and stroke are unhealthy food, lack of physical activity, smoking, and alcohol drinking [1]. A heart attack occurs when the heart's blood circulation is obstructed by arteries plaque build-up. A thrombus in an artery causes a stroke by impeding blood flow to the brain [2]. The symptoms are common to other illnesses and might be confused with indicators of ageing, making diagnosis difficult for practitioners.

Precision prediction and timely identification of cardiac disease are essential for improving patient survival rate. Because of the increased collection of medical data, practitioners now have a great opportunity to promote healthcare diagnosis. ML plays a vital role in many applications like text detection and recognition [3], early prediction [4], power quality disturbance detection [5], truck traffic classification [6], and agriculture [7]. ML has now become an essential tool in the healthcare sector to aid with patient diagnosis. The current methods for predicting and diagnosing cardiac disease are mostly dependent on practitioners' evaluation of a patient's medical history, signs, and physical assessment reports. Nowadays, information about patients with clinical reports is widely accessible in databases in the healthcare field, and it is rising rapidly day by day. In this article, the UCI ML repository's Cleveland HD dataset was utilized for developing the prediction model to heart disease. The machine is trained for learning patterns based on the features that are already present in the dataset. Classification is an effective ML approach for prediction. When properly trained with adequate data, classification is an effective supervised ML method for identifying disease [8]. The primary goal of this work is to employ contemporary ML techniques to construct the healthcare heart disease predictive model. The Cleveland HD dataset was subjected to SVM with radial basis function (RBF) kernel, Gaussian Naive Bayes, logistic regression, LightGBM, XGBoost, and random forest algorithm, and the best performing prediction model for early diagnosis of heart disease was found.

The article "Implementation of a Heart Disease Risk Prediction Model Using Machine Learning" was retracted in 2023. Reasons: unreliable results or conclusions; concerns about the data; concerns about the peer review; concerns about the citations.

## 2. Related Work

Nave Bayes, random forest, PART, C4.5, and multilevel perceptron algorithm-based predictive model accuracy to HD dataset were determined to be in the range of 75.58%–83.17% [9]. Moreover, Nave Bayes algorithm has the highest accuracy as 83.17%, while other algorithms have less than 80% accuracy [9]. Kumar et al. discovered that the Random Woodland ML classifier had an 85 percent precision for cardiovascular disease [10].

Gudadhe et al. [11] described the framework for predicting the heart disease using SVM and obtained the accuracy as 80.41%. Kahramanli and Allahverdi [12] combined fuzzy and cris*p* values in health data and attained accuracy rates of 84.24% to Pima Indian diabetes dataset and 86.8% for the Cleveland HD dataset, respectively. Various ML classification models [13–17] could be used to improve intelligence. Kahramanli and Allahverdi [12] established the artificial and fuzzy-based model to the Pima Indian diabetes dataset and the Cleveland HD dataset and found 84.24% and 86.8% accuracy, respectively.

The article "Implementation of a Heart Disease Risk Prediction Model Using Machine Learning" was retracted in 2023. Reasons: unreliable results or conclusions; concerns about the data; concerns about the peer review; concerns about the citations.

Olaniyi et al. [18] established a prediction model and achieved an accuracy of 85% using feedforward multilayer perceptron (MLP) and 87.5% using SVM on the UCI ML datasets. Polat et al. [19] have employed k-nearest neighbour algorithm and an artificial immune recognition framework and achieved 87% accuracy on the Cleveland dataset. On a Cleveland dataset, Detrano et al. [20] achieved 77% using the logistic regression algorithm. Saw et al. [21] have implemented the improved logistic regression classification model for heart disease dataset. The fast decision tree and C4.5 tree have been employed for HD prediction [22]. As a result of the proposed model's initial phase, trees and features have been extracted. The genetic and fuzzy logic-based approach has been proposed [23] which is a hybrid model to instantly generate the rules using a fitness function, appropriate genetic operators, and a rule encoding method.

In this article, SVM with RBF kernel, Gaussian Naive Bayes, logistic regression, LightGBM, XGBoost, and random forest algorithms were employed to evaluate the classification accuracy on UCI ML repository's Cleveland HD dataset [24]. The data visualization has also been done to illustrate the relationship between the features.

## 3. Materials and Methods

### 3.1. Data

The UCI ML repository's Cleveland HD dataset was used in this investigation [24]. As indicated in Table 1, a subset of 13 attributes were utilized in prediction of heart disease with 303 data instances. Table 1 describes about the attributes and its description that were used in the proposed classification model. The clinical variables that were considered to be essential were given under attribute column in Table 1, and it is chosen based on the chi-square (chi^2^) feature selection method [25]. To develop the heart risk prediction model, the remaining 61 attributes of the dataset were excluded to improve the accuracy of the model. Except for null, all other target values from 1 to 4 were considered as risk of cardiovascular disease for developing the model. The classification model consists of two classes, namely, class 0 and 1. The target values 1 to 4 have been changed as 1 during preprocessing.

### 3.2. Feature Selection

The statistical overview of subset attributes is shown in Table 2 for 303 instances. The count shows us how many nonempty rows are there in a feature. The value of “mean” indicates the feature's average value. The value of “std” reflects the feature's standard deviation. The “min” indicates the feature's minimal value. The 25%, 50%, and 75% are the percentile/quartile of each feature. The maximum value of the attribute is indicated by “max.”

The article "Implementation of a Heart Disease Risk Prediction Model Using Machine Learning" was retracted in 2023. Reasons: unreliable results or conclusions; concerns about the data; concerns about the peer review; concerns about the citations.

Statistical tests will be useful in determining which attributes are having the most powerful relationship with the performance variable. The “SelectKBest” class in Python's scikit-learn library is utilized to choose a distinct attribute in a statistical test set. For nonnegative characteristics in this dataset, the statistical chi-square (chi^2^) test was used to pick 13 of the best features.

### 3.3. Dataset Visualization

The data visualization of features such as gender, chest pain category, and fasting blood sugar level of the Cleveland heart dataset is shown in Figure 1. Males are more likely than females to get heart disease, according to this Cleveland dataset. The majority of individuals with cardiovascular disease experience asymptomatic chest discomfort.

Figure 2 depicts a heat map of the subset attributes, which serves as an instant visual summary. Thalassemia is a genetic disorder that causes people to have low haemoglobin levels than normal. Haemoglobin allows erythrocyte to transmit oxygen.  Figure 3 illustrates the distribution of thalach, chol, trestbps, and people count those who are suffering from cardiovascular disease based on to their age. Cardiovascular disease is quite common in people over the age of 60, as well as adults aged 41 to 60. However, it is uncommon in the 19-year to 40-year-old age category and extremely uncommon in the 0-year to 18-year-old age category.  Figure 4 shows the correlation between attributes such as thalach and chol, age and target, age and ca, thalach and CP, and oldpeak and exang with respect to target.  Figure 5 shows the pair plot that is useful to quickly explore distributions and relationships between the attributes. In adult people, total cholesterol levels < 200 mg/dL are generally preferred. In the range 200-239 mg/dL, 240 mg/dL, and above, borderlines are regarded to be high. A value of <40 mg/dL is measured as a risk factor for HD. A level of 41 mg/dL to 59 mg/dL is considered borderline low. The maximal HDL level that may be measured is 60 mg/dL.

## 4. Proposed Machine Learning Classifiers

To evaluate the heart disease risk prediction, six ML classifiers were used: SVM with RBF kernel, Gaussian Naive Bayes, logistic regression, LightGBM, XGBoost, and random forest.

### 4.1. Support Vector Machine

The SVM [26] classifier with RBF kernel is a function that turns a nonlinear problem into a linear problem in a multidimensional space. The RBF kernel in SVM classification algorithm is defined as

(1) $$\begin{array}{c} K\left(x,x^{\prime }\right)=e^{-\gamma {\left|\left|x-x^{\prime }\right|\right|}^{2}}, \end{array}$$

where ‖*x* − *x*′‖^2^ is the squared Euclidean distance between two feature vectors and *γ* is a scalar.

The article "Implementation of a Heart Disease Risk Prediction Model Using Machine Learning" was retracted in 2023. Reasons: unreliable results or conclusions; concerns about the data; concerns about the peer review; concerns about the citations.

### 4.2. Gaussian Naive Bayes

Gaussian Naive Bayes is the classification algorithm, and here, the 13 features stochastically independent for every class c and the prediction are given as

(2) $$\begin{array}{c} p\left(x_{i}\;\;|\;\;c_{j}\right)=\frac{1}{\sqrt{2\Pi \sigma_{i,j}^{2}}}\;e^{-1/2{\left(x_{i}-\mu_{i,j}/\sigma_{i,j}\right)}^{2}}\text{for }i=1,2,\cdots ,13\text{ and }j=0,1,2,3\&4, \end{array}$$

where *μ*_*i*,*j*_ is the mean and *σ*_*i*,*j*_ is the root-mean square deviation of the dataset.

### 4.3. Logistic Regression

The logistic regression model is expressed as

(3) $$\begin{array}{c} P\left(y=1\;|\;x\right)=p\left(\alpha ,\beta \right)=\frac{e^{\alpha +X^{T}\beta }}{1+e^{\alpha +X^{T}\beta }}, \end{array}$$

where *α* is intercept arguments, *β* is slope argument vector, and *D*_*n*_ = {(*X*_*i*_, *y*_*i*_), *i* = 1, 2, 3, ⋯, *n*} is the independent data size of *n* with 303 data instances.

### 4.4. LightGBM

The LightGBM [27] is a gradient-based boosting approach which makes use of tree-based learning methods. The pseudocode of the algorithm is given below.

### 4.5. XGBoost

XGBoost algorithm is adopted from [28] and the pseudocode of the algorithm is given below.

### 4.6. Random Forest

The random forest [29] constructs multiple decision trees and the pseudocode of the algorithm is given below.

## 5. Results and Discussion

The Cleveland HD dataset is split into training and testing set with a ratio of 80 : 20. The classification model accuracy is evaluated using the performance matrices from confusion matrix and it is expressed as

(4) $$\begin{array}{c} \%\text{Accuracy}=\frac{\text{TP}+\text{TN}}{\text{TP}+\text{TN}+\text{FP}+\text{FN}}\times 100, \end{array}$$

where TP stands for true positive, TN stands for true negative, FP stands for false positive, and FN stands for false negative.  Table 3 gives testing set and training set accuracy in % for all the six classifier models.  Figure 6 depicts the accuracy of all models graphically. Figures 7 and 8 show the confusion matrix and receiver operating characteristic (ROC) curves for all six ML classification models. The validation indicates that the random forest algorithm provides better accuracy in prediction. The test set prediction accuracy of the random forest algorithm is 88.5% with ROC of 0.92 for the selected 13 attributes of the 303 data instances of the UCI ML repository's Cleveland HD dataset. The area under the curve (AUC) is an indicator of a classifier's ability to differentiate among classes and can be used to analyse the receiver operating characteristic (ROC) curve. The greater the AUC, the more accurate the model is at discriminating between favourable and unfavourable classes.

The article "Implementation of a Heart Disease Risk Prediction Model Using Machine Learning" was retracted in 2023. Reasons: unreliable results or conclusions; concerns about the data; concerns about the peer review; concerns about the citations.

## 6. Conclusion

The six ML classification algorithms, namely, SVM with RBF kernel, Gaussian Naive Bayes, logistic regression, LightGBM, XGBoost, and random forest, were applied to UCI ML repository's Cleveland HD dataset, and the prediction model has been developed for cardiovascular disease. The random forest algorithm provides better accuracy as 88.5% followed by SVM, and logistic regression provides 80.32% accuracy for the selected 13 attributes using the chi-square distribution. In this classification model, totally 303 data instances have been used. In future, various heart disease datasets from health data repository can be combined, and the best performing classification model using contemporary machine learning models can be outlined.

## Figures and Tables

**Figure 1:** Visualization of features of the Cleveland heart dataset.

**Figure 2:** Heat map of subset attributes.

**Figure 3:** Distribution of various attributes.

**Figure 4:** Subset attribute correlation.

**Figure 5:** Pair plot.

**Figure 6:** ML classification models—prediction accuracy.

**Figure 7:** Confusion matrix.

**Figure 8:** Performance of classification models—ROC curves.

**Pseudocode 1:** LightGBM.

**Pseudocode 2:** XGBoost.

**Pseudocode 3:** Random forest.

**Table 1:** UCI ML repository's Cleveland heart disease dataset—feature subset [24].

Attribute name	Attribute description
Age	Age in years
Sex	1 denotes male and 0 denotes female
CP	Chest pain type 1, typical angina; type 2, atypical angina; type 3, nonanginal pain; and type 4, asymptomatic
trestbps	Resting blood pressure (in mmHg at entry to the health center)
chol	Serum lipid level in mg/dL
fbs	1 denotes true, i.e., the fasting blood sugar level > 120 mg/dL; 0 denotes false
restecg	Resting ECG results: null, normal; 1, ST-T wave abnormality; and 2, probable or definite left ventricular hypertrophy
thalach	Maximum heart rate achieved
exang	Exercise induced angina (1 = yes; null = no)
oldpeak	ST depression induced by exercise relative to rest
slope	The slope of the peak exercise ST segment (1, 2, and 3): 1, upsloping; 2, flat; and 3, downsloping
ca	Number of major vessels (0-3) colored by fluoroscopy
thal	Thalassemia: 3 = normal, 6 = fixed defect, and 7 = reversible defect

**Table 2:** Statistical outline of subset attributes.

Attributes	Age	Sex	CP	trestbps	chol	fbs	restecg	thalach	exang	oldpeak	slope	ca	thal	target
mean	54.44	0.68	3.16	131.69	246.69	0.15	0.99	149.61	0.33	1.04	1.60	0.66	4.70	0.94
std	9.04	0.47	0.96	17.60	51.78	0.36	0.99	22.88	0.47	1.16	0.62	0.93	1.97	1.23
min	29	0	1	94	126	0	0	71	0	0	1	0	0	0
25%	48	0	3	120	211	0	0	133.5	0	0	1	0	3	0
50%	56	1	3	130	241	0	1	153	0	0.8	2	0	3	0
75%	61	1	4	140	275	0	2	166	1	1.6	2	1	7	2
max	77	1	4	200	564	1	2	202	1	6.2	3	3	7	4

The article "Implementation of a Heart Disease Risk Prediction Model Using Machine Learning" was retracted in 2023. Reasons: unreliable results or conclusions; concerns about the data; concerns about the peer review; concerns about the citations.

**Table 3:** Classification model—prediction accuracy.

Machine learning classifier	Accuracy	
	Training set (80%)	Test set (20%)
SVM	92.56	80.32
Gaussian Naive Bayes	86.77	78.68
Logistic regression	85.95	80.32
LightGBM	98.76	77.04
XGBoost	99.58	73.77
Random forest	100	88.5

## Data Availability

The dataset is available in publicly accessible database.
